# Effects of a Chlorogenic Acid-Containing Herbal Medicine (LAS^NB^) on Colon Cancer

**DOI:** 10.1155/2021/9923467

**Published:** 2021-08-20

**Authors:** Yanchu Li, Rong Pu, Lu Zhou, Dan Wang, Xianyong Li

**Affiliations:** ^1^Oncology Department, West China Hospital of Sichuan University, Chengdu, China; ^2^Oncology Department, Chengdu Fuxing Hospital, Chengdu, China; ^3^Research Department, Chengdu Fuxing Hospital, Chengdu, China

## Abstract

**Background:**

Plant polyphenols, which contain phenolic acids such as chlorogenic acid (CGA), can be used for the treatment of gastrointestinal cancer and have gained increasing attention in recent years. In this study, we explored a novel CGA-containing herbal medicine named LAS^NB^, which was extracted from *Lonicera japonica* Thunb., *Agrimonia eupatoria* L., and *Scutellaria barbata* D.Don.

**Methods:**

CGA in LAS^NB^ was analyzed using high-performance liquid chromatography (HPLC). The biological functions and molecular mechanisms of LAS^NB^ were investigated in colon cancer cell lines (HCT116, HCT15, and CT26), a normal colon cell line (NCM460), and a CT26 xenograft model. To assess safety, hematological toxicity and pathology of the liver, kidney, and lung were evaluated.

**Results:**

LAS^NB^ suppressed HCT116, HCT15, and CT26 colon cancer progression by inhibiting proliferation capacity, promoting cell apoptosis, and suppressing cell migration both in vitro and in vivo. Investigation into the underlying molecular mechanism indicated that LAS^NB^ suppressed the activation of receptor tyrosine kinase- (RTK-) MEK-ERK and NF-*κ*B pathways. With regard to safety, slight interstitial vascular congestion in the lung was observed, but no severe pathological or hematological toxicity was detected.

**Conclusions:**

We found that LAS^NB^ suppressed the progression of colon cancer via the RTK-MEK-ERK and NF-*κ*B pathways, with no severe toxicity observed. Therefore, LAS^NB^ has the potential to be used as a supplementary herbal medicine for the treatment of colon cancer.

## 1. Introduction

Natural products, such as herbal extractive products, have historically made an important and major contribution to pharmacotherapy, especially for cancer diseases [1, 2]. According to the National Central Cancer Registry of China (NCCR), colon cancer is one of the most common cancers and presents an upward trend in age-standardized mortality rates [3, 4]. Several studies have focused on the effect of herbal medicines (HMs) in palliative care, revealing that HMs may have immunomodulatory effects and improve the quality of life and survival time of cancer patients [5, 6]. Recently, phenolic acids have gained considerable attention due to their various biological and pharmacological effects. Indeed, polyphenol-rich extracts from *Pleurotus eryngii*, green tea, and green coffee have shown promising effects in the treatment of inflammatory disease and colon cancer by suppressing p-I*κ*B protein expression, inhibiting NF-*κ*B and I*κ*B mRNA expression, and arresting the cell cycle at the G2/M phase [7–10].

Chlorogenic acid (CGA) is one of the most widely available acids among phenolic acid compounds and has been considered for use in the treatment of gastrointestinal disease. The colon plays a pivotal role in CGA metabolism, and the majority of CGA (approximately 70%) is cleaved in the lower gastrointestinal tract by gut microflora; this results in the release of free CGA and additional microbial metabolites, including 3-phenylpropionic acid (3-PPA) and benzoic acid (BA), with various biological effects [11, 12]. CGA is also known as 5-dicaffeoylquinic acid (5-CQA) according to the guidelines of the International Union of Pure and Applied Chemistry (IUPAC). CGA has several properties that make it suitable for use as a treatment option. Indeed, CGA possesses antioxidant, antibacterial, hypoglycemic, lipid-lowering, anticardiovascular, and immunomodulatory abilities [13, 14], as well as the ability to suppress tumorigenesis [15, 16] via its effects on apoptosis-associated genes [17] and cell-cycle arrest [18, 19]; however, the underlying mechanisms have not been studied extensively [19, 20]. In the current study, we sought to identify a CGA-containing functional herbal compound.

To this end, we formulated a novel CGA-containing herbal compound extracted from *Lonicera japonica* Thunb., *Agrimonia eupatoria* L., and *Scutellaria barbata* D.Don (denominated LAS^NB^) and aimed to identify as well as explore its function and molecular mechanism in the context of colon cancer progression.

## 2. Materials and Methods

### 2.1. Cell Lines and Culture

CT26, HCT116, and HCT15 colon cancer cell lines and NCM460 normal colon cell line were used in this study. The CT26 cell line was purchased from the Shanghai Institutes for Biological Sciences. HCT116, HCT15, and NCM460 cell lines were donated by the State Key Laboratory of Biological Treatment at Sichuan University. All cells were cultured in 10% fetal bovine serum (FBS) in DMEM (Thermo Scientific HyClone, USA) and supplemented with 1% penicillin and streptomycin (Thermo Scientific HyClone). The four cell lines were cultured at 37.0°C in an atmosphere of 5% CO_2_.

### 2.2. Herbal Materials and Preparation of LAS^NB^

LAS^NB^ is a HM prescription for the treatment of colon cancer and was developed by the Pharmaceutical Department of Chengdu Fuxing Hospital. LAS^NB^ was prepared mainly from extracts of 440 g dry flower of *Lonicera japonica* Thunb. (Chinese name: Jin Yinhua; habitat: Sichuan, China), 440 g dry cauline leaf of *Agrimonia eupatoria* L. (Chinese name: Xian Hecao; habitat: Gansu, China), and 440 g dry whole plant of *Scutellaria barbata* D.Don (Chinese name: Ban Zhilian; habitat: Jiangsu, China). The herbs were mixed and pulverized into a coarse powder and soaked in 0.5% hydrochloric acid at 26°C for 2 h. The solution was concentrated and adjusted to pH 10 with strong ammonia water. The precipitate was discarded by centrifugation at 3500 rpm for 25 min, before being extracted three times with *n*-butanol. The extract was dried in rotary evaporators and a vacuum drying chamber; the dried fractions were stored at 26°C in a dryer. The yield of LAS^NB^ extract obtained was 36.7%.

### 2.3. CGA Analysis of LAS^NB^

High-performance liquid chromatography (HPLC) was used to identify CGA in LAS^NB^. LAS^NB^ extract (10 *μ*L sample; 1 mg/mL) and CGA standard reference were injected into the HPLC system (Waters 2695 and Waters 2996 Diode Array Detector, USA) and separated on a C18 ODS column (Hypersil ODS2 4.6 × 250 mm, 5 *μ*m; ELITE, China) with gradient elution for 15 min (acetonitrile 0.4%: phosphoric acid solution = 13 : 87) at 25°C. The flow rate was 1.0 mL/min, and detection was performed at 327 nm.

### 2.4. MTT Assay

The effect of LAS^NB^ on cell viability was assessed using a MTT assay (Sigma-Aldrich, USA). Colon cancer cells (CT26, HCT15, and HCT116) and normal colon cells (NCM460) were seeded (5 × 10^3^ cells/well) in 96-well plates and exposed to 0.625–10.0 mg/mL LAS^NB^. After 24 h incubation, 20 *μ*L of 5 mg/mL MTT solution was added to each well, and the plate was further incubated at 37°C for 4 h. Thereafter, the medium was aspirated, and 200 *μ*L of DMSO was added to each well [21]. After the formazan crystals had dissolved, the absorbance was determined spectrophotometrically at 492 nm on an INFINITE F50 microplate reader (TECAN, Austria).

### 2.5. Crystal Violet Assay

CT26, HCT15, and HCT116 colon cancer cells were seeded in 24-well plates (2 × 10^3^ cells/well) and incubated for 24 h. Following incubation, the cells were treated with or without LAS^NB^ at different concentrations (1.25, 2.5, 3.0, and 4.0 mg/mL) for 5 days. After fixation with 4% paraformaldehyde for 30 min, the cells were stained with crystal violet solution for 2 h. Photographs of the colonies were obtained manually after washing with phosphate-buffered saline (PBS).

### 2.6. Cell Scratch Assay

Cell migration ability was quantitated using a cell scratch assay. Approximately 2 × 10^5^ cells were aliquoted into each well of a 6-well plate, and a microscope was used the following day to confirm that each well was coated with cells. A 1 mL pipette tip was used to scratch the cells from the well, and the plates were washed three times with PBS to remove the displaced scratched cells. Cells were exposed to LAS^NB^ at a concentration of 3.0/4.0 mg/mL. Cells were cultivated simultaneously in an incubator at 37°C and 5% CO_2_. Images of the samples were captured at 0, 24, 48, and 72 h using a Nikon TS100 microscope (Nikon, Japan). The procedure was repeated three times.

### 2.7. Flow Cytometry Assay

HCT116, CT26, and HCT15 cell lines (5 × 10^5^ cells/well) were seeded in 6-well plates, and the cells were exposed to LAS^NB^ (IC50 = 2.98 mg/mL, 3.15 mg/mL, and 2.46 mg/mL, respectively) for 24 h. The cells were then trypsinized and resuspended to obtain single cell suspensions. For apoptosis analysis, cells were stained with fluorescein isothiocyanate-conjugated Annexin V and propidium iodide (apoptosis detection kit; Keygen, China) for 10 min in the dark, as recommended by the manufacturer. Samples were tested using a BD LSR Fortessa flow cytometer (Becton, Dickinson and Company, USA) and analyzed using FlowJo V10.0 (Becton, Dickinson and Company, Ashland, USA). The experiment was repeated three times.

### 2.8. Western-Blot Assay

The expressions of EGF (Abcam, ab184265, 1 : 1000), VEGF (Abcam, ab32152, 1 : 1000), NF-*κ*B p65 (Beyotime, AN365, 1 : 1000), NF-*κ*B p50 (Abcam, ab32360, 1 : 1000), p-ERK (Beyotime, AF1891, 1 : 1000), T-ERK (Beyotime, AF1051, 1 : 1000), and TGF-*β* (Beyotime, AF0297, 1 : 500) were measured in CT26 tumor tissue and CT26 and HCT15 cell lines. Protein concentrations were determined using a BCA kit (Beyotime, China). Protein samples were resolved by SDS-PAGE and transferred to polyvinylidene fluoride membranes (Merck Millipore, USA). Immunoblotting was performed overnight at 4°C. The membranes were then washed three times with TBST and incubated with the corresponding secondary antibodies (1 : 5000) at room temperature for 2 h. Following incubation, the membranes were washed three times with TBST, and the proteins were visualized using an enhanced chemiluminescence assay kit (Beyotime, China). Images were captured using the G: BOX ChemCR system (Syngene, UK).

### 2.9. CT26 Xenograft Model and Treatment

Female SPF-BALB/c mice weighing 21.0 ± 1.2 g were obtained from the Institute of Experimental Animals of Sichuan People's Hospital (Chengdu, China). The animal study was approved by the Animal Care and Use Committee. For each mouse, 4% chloralic hydras were used at a dose of 0.1 ml/10 g. CT26 cells (1 × 10^6^ cells/mouse) were transplanted to the right side of the back. Sixteen tumor-bearing mice were divided into two groups (*n* = 8 each). Saline was administered to the control group, while 2.61 g/kg LAS^NB^ was administered to the experimental group by oral gavage. The tumor volume and weight were recorded at 3-day intervals. The tumor volume was calculated using the following formula: volume (mm^3^) = width^2^ × length/2.

### 2.10. Hematoxylin-Eosin (HE) Staining Assay

Liver, lung, and kidney tissues were dissected from implanted mice, fixed in 10% buffered formalin for 24 h, and embedded in paraffin. Paraffin-embedded blocks were prepared, and 5 *μ*m thick sections were cut and stained with hematoxylin-eosin (HE) for histological examination. Images were acquired using an Olympus BX50 (Olympus, Japan).

### 2.11. Hematology Toxicity Assay

Blood samples were collected from the implanted mice by eyeball extirpation, and clear serum samples were prepared. Liver and kidney function tests and blood tests were performed using a COBAS INTEGRA 400 Plus (Roche, Switzerland) Chemistry Analyzer and XT-2000i Blood Cell Analyzer (SYSMEX, Japan), respectively.

### 2.12. Immunohistochemistry Assay

Tissues were fixed in 10% buffered formalin and embedded in paraffin. Paraffin sections of tumor tissues were prepared, dewaxed by dimethyl-benzene, and hydrated with different concentrations of ethanol (100%, 95%, 85%, 70%, and 50%). Subsequently, the following steps were performed: blocking of endogenous peroxidase activity in 3% H_2_O_2_ solution, unmasking of the antigenic epitope with citrate buffer, addition of blocking buffer for blocking, and addition of primary antibody VEGF (Bioss, BS1665R, 1 : 1000), CD34 (Bioss, BS5085R, 1 : 1000), and EGF (Bioss, BS1007R, 1 : 1000) and a secondary antibody (horseradish peroxidase-labeled goat rabbit IgG [H + L]; Beyotime, A0208). Finally, DAB substrate solution was applied to reveal the staining. Images were acquired using a Motic BA400 microscope (Motic, China).

### 2.13. Statistical Analysis

Data are expressed as means, and *t*-tests were performed for statistical analysis using GraphPad Prism 8.0. Statistical significance was set at *p* < 0.05.

## 3. Results

### 3.1. LAS^NB^ and CGA Analysis

To confirm the stability of LAS^NB^, the chromatographic fingerprint (CF) similarity of three batches of LAS^NB^ fractions was compared with the generated chromatographic control fingerprint (GCCF). According to the results, the CF similarity of the three batches of LAS^NB^ fractions was up to 0.808 (>0.8) compared with their GCCF (Figure 1(a)). The chromatographic peak was identified by comparing the retention time with that of chlorogenic acid reference (purity: 99.39%, product number: A0022, Chengdu Must Bio-technology Co., Ltd., China). According to the result, CGA in the LAS^NB^ sample (Sample, S) was detected at the peaks of 6.204 and 6.628 min, which is consistent with the peak of the CGA reference (Reference, R) (Figure 1(b)). According the HPLC analysis, the purity of chlorogenic acid is 1.73% in the LAS^NB^ extract sample.

### 3.2. LAS^NB^ Inhibits Proliferation of Colon Cancer Cell Lines and Promotes Apoptosis

MTT and colony formation assays were performed to investigate the anticancer function of LAS^NB^ on the short- and long-term proliferation capacity after LAS^NB^ treatment. The results of the MTT assay showed that the short-term proliferative capacity of HCT116, CT26, HCT15, and NCM460 cells was inhibited by 88.45% ± 2.01%, 77.20% ± 3.97%, 88.17% ± 4.57%, and 15.27% ± 1.74%, respectively (Figure 2(a)), with dose-dependent effects. However, LAS^NB^ only slightly influenced the NCM460 normal colon cells, with an inhibition rate <15.0%. According to the results, the IC50 of LAS^NB^ against HCT116, CT26, and HCT15 cells was 2.98 mg/mL, 3.15 mg/mL, and 2.46 mg/mL, respectively. The morphology of CT26 and HCT116 cells changed to narrow (Figure 2(b)). The results of the colony formation assay showed that the long-term proliferation capacity was suppressed in CT26, HCT116, and HCT15 (Figure 2(c)).

Next, we investigated the effects of LAS^NB^ on the induction of apoptosis. As shown in Figure 2(d), the proportion of annexin V(+)/PI −), annexin V(+)/PI(+), and annexin V(−)/PI(+) apoptotic/dead cells increased after LAS^NB^ treatment. In CT26, HCT15, and HCT116 cell lines, the early-apoptosis percentages were 54.58% ± 4.01% (*p* < 0.005^*∗∗∗*^), 13.83% ± 2.76% (*p* < 0.05^*∗*^), and 14.97% ± 3.58% (*p*=0.06), respectively, the late-apoptosis percentages were 10.88% ± 1.49% (*p* = 0.15), 6.18% ± 1.83% (*p* < 0.05^*∗*^), and 3.49% ± 1.28% (*p*=0.32), respectively, and the cell death percentages were 1.12% ± 0.05% (*p*=0.91), 15.30% ± 0.68% (*p* < 0.005^*∗∗∗*^), and 5.29% ± 0.57% (*p* < 0.05^*∗*^), respectively.

### 3.3. LAS^NB^ Inhibits Cancer Cell Migration

To investigate the effect of LAS^NB^ on cancer cell migration, differences in the scratch cell areas of CT26 and HCT116 cells within 72 h were observed. According to the results, the relative scratch width [2] of the LAS^NB^ group was significantly wider than that of the control group. In the high-dose LAS^NB^ group, it was difficult to observe cell migration; in contrast, the scratch damage area of the control group was filled with migrated CT26 and HCT116 cells. These data indicated that LAS^NB^ inhibited cell migration in a concentration-dependent manner (Figure 2(e)).

### 3.4. LAS^NB^ Inhibits Tumor Progression in CT26 Tumor-Bearing Mice

The tumor weight and volume of CT26 tumor-bearing mice in the LAS^NB^ group (dose = 2.61 g/kg) were significantly reduced compared with those in the control group (Figure 3(a)). The inhibition rates of tumor weight and volume were 68.35% (2.85 ± 0.89 g vs. 4.69 ± 1.17 g) and 47.68% (1894.28 ± 735.91 mm^3^ vs. 4361.97 ± 1107.34 mm^3^), respectively (Figures 3(b) and 3(c)). As shown in Figure 4(a), cell apoptosis was observed, and integrated optical density (IOD) of EGF, VEGF, and CD34 expression in the LAS^NB^ group was 0.0948 ± 0.0173, 0.0177 ± 0.0103, and 0.1535 ± 0.0173, respectively, compared with 0.1620 ± 0.0143, 0.0586 ± 0.0095, and 0.2355 ± 0.0197 in the control group, respectively (Figure 4(b)). The TUNEL-positivity rate in the LAS^NB^ group was 47.50% ± 17.04% compared with 8.50% ± 7.96% in the control group (Figure 4(b)).

To further elucidate the underlying mechanisms of LAS^NB^, we evaluated the downstream kinase of RTK-MAPK and NF-*κ*B pathway expression by western blotting. According to the results, both expression rates of RTKs, such as EGF, VEGF, and TGF-*β*, were prohibited in vitro and in vivo by LAS^NB^, as was the expression of key proteins involved in the MAPK and NF-*κ*B pathways, such as *p*-ERK, NF-*κ*B p65, and NF-*κ*B p50 (Figure 4(c)). In summary, the working model describes that LAS^NB^ could suppress the proliferation and antiapoptosis of colon cancer by acting on RTK signals, the canonical MAPK cascade, and the NF-*κ*B pathway.

### 3.5. Toxicity Assessment in Tumor-Bearing Mice

Hematological and pathological analyses were performed. In the hematology assay, the serum levels of alanine aminotransferase (ALT) and aspartate aminotransferase [22] were measured as indices of hepatic function, the levels of blood urea nitrogen (BUN) and creatinine served as indexes of renal function, and the proportion of white blood cells (WBC), red blood cells (RBC), and blood platelets (PLT) as well as the lymphocyte ratio (LYM%) served as indices of the routine blood test [23]. According to the results, no hematological toxicity over Grade II (CTCAE 3.0) was observed compared with the control group (Figure 5(a)). In addition, no kidney or liver pathology was observed, except for slight interstitial vascular congestion in the lungs in LAS^NB^ group (Figure 5(b)). Thus, the data indicated that LAS^NB^ treatment of tumor-bearing mice was safe.

## 4. Discussion

Recently, surgery, chemotherapy, target therapy, and immunotherapy have been considered the main treatment methods, either alone or in combination, to suppress cancer progression. In the meantime, HMs have gained more attention for the maintenance and palliative care treatment for late-stage patients. HMs, which have been used for thousands of years, play an important role in the treatment of various diseases, including cancer [24, 25]. In the area of cancer, over the time frame from around the 1940s to the end of 2014, 175 small molecules from natural products were approved as sources of new drugs; 131(75%) are other than synthetic, with 85 (49%) actually being either natural products or directly derived therefrom [26]. Nowadays, modern biological methods are used to explore the pharmacological effects of HMs, and many studies have shown the complexity of HM compounds. Indeed, HMs treat diseases via multiple synergistic effects on multiple components with multiple targets, such as by regulating angiogenesis, inducing cancer cell differentiation or apoptosis, and enhancing cytotoxic function and immunity regulation, compared with the effects of chemical drugs [24, 27, 28]. For instance, astragalus-based HM enhances the efficacy of platinum-based chemotherapy and improves platinum-derived toxicities for late-stage non-small-cell lung carcinoma (NSCLC) [29]. Moreover, KIOM-C and *Ganoderma lucidum* have been shown to abrogate the metastatic potential of malignant HT1080 cells and reduce ovarian cancer cell growth by reducing MMP activity via the suppression of NF-*κ*B activation and downregulation of VEGF expression, respectively [30–32]. Commonly known, NF-*κ*B is responsible for some important genes' regulation, including survival, inflammation, and immune responses, and its aberrant activation has been observed in several cancer types and is known to contribute to aggressive tumor growth and resistance to therapeutic treatment [33].

In addition, phenolic acids, which are essential plant polyphenols and the main active ingredients in Flos Lonicerae extract, possess strong antibacterial, antioxidant, and antiviral properties that are involved in treating gastrointestinal diseases [34–37]. Furthermore, CGA, which is an important phenolic acid, acts as a principal bioactive phytoconstituent, with potential anticancer functions. In previous studies, CGA was shown to induce the Nrf2/ARE antioxidant system, which synthesizes antioxidant and phase II detoxifying enzymes to eliminate oxidative stress damage caused by various injury-related factors in hepatic cells [38, 39]. CGA was also shown to protect the JB6 cell line against environmental carcinogen-induced carcinogenesis by upregulation of cellular antioxidant enzymes and suppression of ROS, NF-*κ*B, and MAPK pathways [22]. Moreover, CGA has also been shown to block the migration capacity of U-87 glioma cells [40].

Few studies have investigated the effects of CGA-based medicine against colon cancer. However, Hou et al. reported that CGA could induce ROS production and inhibit cell viability in human colon cancer cells by influencing cell cycle and ERK inactivation [19]. Therefore, this study was designed to explore the antitumor effects and molecular mechanisms of a novel CGA-based compound medicine. As expected, LAS^NB^ had a positive role in inhibiting the growth of colon cancer both in vitro and in vivo, as demonstrated by MTT, scratch assay, flow cytometry, HE, IHC, and TUNEL assays.

According to our in vitro results, LAS^NB^ inhibited the proliferation and migration capacity of HCT116, HCT15, and CT26 colon cancer cell lines. The inhibition rate of proliferation at the high dose was 77.20%–88.45%, while that of the low dose was 4.85%–22.61%. In contrast, in vivo, CT26-bearing tumor progression was suppressed, and the inhibition rates of the tumor weight and volume reached 68.35% and 47.68%, respectively. Furthermore, in previous studies, RTK cytokines and the MAPK and NF-*κ*B pathways were involved in the regulatory network of cancer progression. Previous studies have indicated that NF-*κ*B is a significant mediator and plays a key function in regulating the human immune system, which is associated with cancer, diabetes, and rheumatoid arthritis [41]. In this study, in order to detect the mechanisms of LAS^NB^, MAPK and NF-*κ*B pathway-related cytokines and key proteins, such as VEGF, EGF, CD34, TGF-*β*, ERK, MEK, and NF-*κ*B P65/50, were evaluated. The results showed that both expression rates of RTKs (EGF, VEGF, and TGF-*β*) were prohibited in vitro and in vivo, as was the expression of key proteins involved in the MAPK and NF-*κ*B pathways (*p*-ERK, NF-*κ*B p65, and NF-*κ*B p50). These results were in accordance with pharmacological effects of LAS^NB^. Thus, consolidating the previous data, the agents that can modulate deregulated RTK-MEK-ERK and NF-*κ*B activation have a great potential for both the prevention and treatment of colon cancer.

In addition, the safety of LAS^NB^ in tumor-bearing mice was also proven, as this treatment did not exacerbate adverse hematological and pathological effects. Thus, LAS^NB^ is an effective and safe preparation method as a supplementary treatment.

## 5. Conclusions

The novel CGA-based compound medicine LAS^NB^ has the potential to function as a therapeutic and useful supplementary medicine against colon cancer.

## Figures and Tables

**Figure 1:** HPLC analysis. (a) Chromatographic fingerprint of the three batches of LAS^NB^ and the generated chromatographic control fingerprint (S_1_, S_2_, and S_3_: three batches of LAS^NB^; FP: GCCF). (b) Peak 1 represents chlorogenic acid (CGA) in CGA reference (R), and peak 2 represents CGA at 6.204 and 6.628 min in the LAS^NB^ sample (S), consistent with the CGA reference (S) LAS^NB^ sample; R: CGA reference.

**Figure 2:** (a) MTT assay. 24 h after exposing CT26, HCT15, HCT116, or MCN460 cells to LAS^NB^. LAS^NB^ inhibited cell proliferation in a concentration-dependent manner and had limited effects on NCM460 cells. (b) Changes in the morphology of CT26 and HCT116 cells after 24 h LAS^NB^ treatment. (c) Crystal violet assay: CT26, HCT15, and HCT116 cells were treated with LAS^NB^, and cell viability was inhibited in a concentration-dependent manner. (d) FCM assay. LAS^NB^ promoted cell apoptosis after 24 h LAS^NB^ treatment (dose = 2.979 mg/ml, 3.145 mg/ml, and 2.455 mg/ml for CT26, HCT15, and HCT116 cells, respectively). (e) Scratch width in the different groups; CT26 (E1) and HCT116 (E2) groups were observed at 0, 24, 48 h, and 72 h, respectively. Magnification, 40x; ^∗^*p* < 0.05, ^∗∗^*p* < 0.01, and ^∗∗∗^*p* < 0.005.

**Figure 3:** Tumor volume and weight of control and LAS^NB^ groups. The tumor volume and weight in the LAS^NB^ group were reduced compared with those in the control group; ^*∗*^*p* < 0.05, ^*∗∗*^*p* < 0.01, and ^*∗∗∗*^*p* < 0.005, respectively.

**Figure 4:** Control and LAS^NB^ xenograft models. (a) Hematoxylin-eosin staining assay results are shown. Compared with the control group, the LAS^NB^ group showed increased colon cell apoptosis. (b) CD34, EGF, and VEGF expression and TUNEL-positive cells were assessed by immunohistochemistry in the tumor microenvironment. Magnification, 400x (*p* < 0.05). (c) Western blot results are shown. The expression of RTK kinase (EGF and VEGF), NF-*κ*B proteins (NF-*κ*B p65, NF-*κ*B p50, and TGF-*β*), and MAPK (p-ERK and t-ERK) in the xenograft model (C1), CT26 cells (C2), and HCT15 cells (C3). ^∗^*p* < 0.05, ^∗∗^*p* < 0.01, and ^∗∗∗^*p* < 0.005.

**Figure 5:** Hematological toxicity and pathology. No hematological toxicity over Grade II (CTCAE 3.0) was observed in the LAS^NB^ group compared with the control group. Slight interstitial vascular congestion in lung was observed in the LAS^NB^ group. In addition, no pathological change was found in the kidney and liver in the LAS^NB^ group. (a) Routine blood test and liver and kidney function test. For liver and kidney functions, the levels of AST, ALT, BUN, and creatinine were 115.18 ± 21.84 U/l (0–80 U/l), 35.28 ± 4.68 U/l (0–77 U/l), 8.59 ± 1.30 mmol/l (2.8–11.9 mmol/l), and 39.90 ± 4.22 *μ*mol/l (10–80 *μ*mol/l) in the LAS^NB^ group compared to 126.30 ± 23.68 U/l, 33.52 ± 2.62 U/l, 8.39 ± 0.59 mmol/l, and 36.84 ± 3.41* μ*mol/l in the control group, respectively (*p* > 0.05). For routine blood tests, the WBC, RBC, PLT, and LYM% were 2.57 ± 1.34 × 10^9^/l (0.8–6.8 × 10^9^/l), 7.58 ± 0.26 × 10^12^/l (6.36–9.42 × 10^12^/l), 1150.80 ± 149.82 × 10^9^/l (450–1590 × 10^9/^l), and 74.18 ± 6.32 (55.8%–90.6%) in the LAS^NB^ group compared to 3.62 ± 2.47 × 10^9^/l, 7.86 ± 0.30 × 10^12^/l, 1293.60 ± 162.00 × 10^9^/l, and 73.68% ± 7.55% in the control group, respectively (*p* > 0.05). (b) HE staining of the lung, liver, and kidney tissues.

## Data Availability

No data were used to support this study.
